# Efficient Parallel Video Processing Techniques on GPU: From Framework to Implementation

**DOI:** 10.1155/2014/716020

**Published:** 2014-03-16

**Authors:** Huayou Su, Mei Wen, Nan Wu, Ju Ren, Chunyuan Zhang

**Affiliations:** School of Computer Science and Science and Technology on Parallel and Distributed Processing Laboratory, National University of Defense Technology, Changsha, Hunan 410073, China

## Abstract

Through reorganizing the execution order and optimizing the data structure, we proposed an efficient parallel framework for H.264/AVC encoder based on massively parallel architecture. We implemented the proposed framework by CUDA on NVIDIA's GPU. Not only the compute intensive components of the H.264 encoder are parallelized but also the control intensive components are realized effectively, such as CAVLC and deblocking filter. In addition, we proposed serial optimization methods, including the multiresolution multiwindow for motion estimation, multilevel parallel strategy to enhance the parallelism of intracoding as much as possible, component-based parallel CAVLC, and direction-priority deblocking filter. More than 96% of workload of H.264 encoder is offloaded to GPU. Experimental results show that the parallel implementation outperforms the serial program by 20 times of speedup ratio and satisfies the requirement of the real-time HD encoding of 30 fps. The loss of PSNR is from 0.14 dB to 0.77 dB, when keeping the same bitrate. Through the analysis to the kernels, we found that speedup ratios of the compute intensive algorithms are proportional with the computation power of the GPU. However, the performance of the control intensive parts (CAVLC) is much related to the memory bandwidth, which gives an insight for new architecture design.

## 1. Introduction

Video encoding plays an increasingly larger role in the multimedia processing community, which aims to reduce the size of the video sequence by exploiting spatial and temporal redundancy, as well as keeping the quality as good as possible. H.264/AVC [1] is currently the widely used video coding standard, which constitutes the basis of the emerging High Efficiency Video Coding (HEVC) [2]. It achieves about 39% and 49% bit-rate saving over that of MPEG-4 and H.263, respectively [3, 4]. The high compression efficiency is mainly attributed to several introduced new features, including variable block-size motion compensation, multiple reference frames, quarter pixel motion estimation, integer transform, in-the-loop deblocking filtering, and advanced entropy coding [5–8]. These new features imply that more computational power is needed for H.264 encoder [9]. It is almost impossible to achieve real-time High-Definition (HD) H.264 encoding in serial programming technologies, which restricts its usage in many areas [10–13]. In order to satisfy the requirement of real-time encoding, many research works focused on hardware-based encoders design [14–17]. Though high efficiency can be gained, dedicated ASIC designs are inflexible, time consuming, and expensive.

Due to the high peak performance, high-speed bandwidth, and efficient programming environments, such as NVIDIA's CUDA [18] and OpenCL [19], GPU has been at the leading edge of high performance computing era. Recently, many researchers are attracted to the topic of parallelizing video processing with multicore or many-core architecture, especially on the GPU-based systems [8–12, 20–27]. However, most of the research has mainly focused on accelerating the computational components, such as the motion estimation (ME) [12, 21, 22], motion compensation [10], and intraprediction [23]. For the irregular algorithms, such as deblocking filter and Context-based adaptive variable-length code (CAVLC), research about these aspects is seldom [24]. To the best of our knowledge, there is no research about GPU-based CAVLC, except our work [28]. There are several disadvantages by only accelerating some parts of video encoder. On the one hand, for each frame, the data size transferred between CPU and GPU will be very huge. For example, when offloading the ME and transform coding to GPU only, the data size of the input frame, the quantized coefficients, and the auxiliary information are more than 30 MB for 1080 p video format. On the other hand, after parallelizing the compute intensive parts of the encoder, the control intensive algorithms occupy a larger fraction of execution time [29]. Though NVIDIA provides a GPU-based encoder library, the detailed information is insufficient, let alone open source. In this paper, we focused on developing a GPU-based parallel framework for H.264/AVC encoder and the efficient parallel implementation. The main contributions of this paper are as follows.

After carefully reviewing and profiling the program, we proposed a fully parallel framework for H.264 encoder based on GPU. We introduced the loop partition technology to divide the whole pipeline into four steps (ME, intracoding, CAVLC, and deblocking filter) in terms of frame. All the four components are offloaded to GPU hardware in our framework. The CPU is only responsible for some simple transactions, such as I/O process. In order to improve the memory bandwidth efficiency, array of structure (AOS) to structure of array (SOA) transformation is performed. The transformed small and regular structures are more suitable for taking the advantage of coalesced accessing mechanism. In addition, the proposed framework exploits the producer-consumer locality between different parts of the encoder, which avoids unnecessary data copy between CPU and GPU.

For the compute intensive component motion estimation, a scalable parallel algorithm has been proposed targeting massively parallel architecture, named multiresolutions multiwindows (MRMW) motion estimation. It calculates the optimal motion vector (MV) for each macroblock (MB) through several steps. Firstly, the original input frame and reference frame are concentrated into small resolution ones. Accordingly, there is a concentrated MB in the dedicated frame corresponding to the normal MB in the original frame. Secondly, based on the concentrated lower resolution frames, a full search in an assigned window space is performed for each concentrated MB and it produced a primary MV. Finally, a refinement search for the MBs of the original frame will be performed; the search window is centered with the produced MV in the second step.

In order to overcome the limitations from the irregular components, a direction-priority deblocking filter [30] and a component-based CAVLC parallel schemes have been proposed. The GPU-based deblocking filter reserves the result data into global memory, which serves as the reference frame for the next frame. In order to further enlarge the parallel degree, based on the direction-priority method, a novel schedule strategy based on [24] is proposed. The proposed CAVLC relieves the data dependence and reduces the amount of data copy back to CPU significantly. Overall, the proposed parallel methods can not only improve the performance of the tools but also reduce the data transferred between host and device.

Based on the multislice technology, a multilevel parallel method is designed for intracoding to explore the parallelism as much as possible [31]. The proposed parallel algorithm improves the parallelism between 4 × 4 blocks within a MB by throwing off some insignificant prediction modes. By partitioning a frame into multislices, the parallelism between MBs can be exploited. In addition, a multilevel parallel scheme was presented to adapt the parallel granularity of different stage of the intracoding.

In summary, we proposed an efficient parallel framework for H.264 encoder based on massively parallel architecture. Not only the compute intensive parts but also the control intensive components are ported to GPUs. Several optimizations are introduced to enlarge the parallelism or improve the bandwidth efficiency, which are the two most important factors impacting the performance of a GPU-based application. Our implementation can satisfy the requirement of real-time HD encoding of 30 fps, while the value of PSNR only reduced from 0.14 to 0.77 dB.

The rest of this paper is organized as follows.  Section 2 is the related work.  Section 3 presents the proposed the efficient parallel H.264 encoder framework. We describe the proposed MRMW algorithm and its implementation with CUDA in Section 4. In Section 5, we discuss the efficient parallelization of the control intensive components. A comprehensive performance evaluation is performed in Section 6. Finally, a conclusion is drawn in Section 7.

## 2. Related Work

At the beginning, motion estimation researches mainly focused on designing optimized algorithms to reduce the computational complexity. Cheung and Po [32] proposed a cross-diamond search algorithm to reduce the search space. In [5], it presented an unsymmetrical-cross multi-hexagon-grid search method to simplify the ME, which can save about 90% of computation compared with the traditional full search algorithm. In the last decade, with the widespread usage of the parallel processors, many researchers are attracted to the field of parallel video processing. A discussion about the parallel methods for video coding was presented in [33], including the hardware and software methods. In [34], the authors implemented a MB-based parallel decode on CELL processor, which can achieve real-time decoding performance. Huang et al. [3] discussed how to optimize the data transfer between host and device when designing the parallel scalable video coding with CUDA. Marth and Marcus [35] presented a parallel x264 [36] encoder with OpenCL.

A large amount of publications reported the GPU-based motion estimation, including using 3D graphic libs and high level programming models [12, 20, 22, 27]. These researches mainly focused on scheduling the search algorithm to explore the parallelism. Kung et al. proposed a block based parallel ME [20], which increased the parallel degree by rearranging the processing order of 4 × 4 blocks. In [12], the authors divided ME algorithm into five fine-granularity steps, so that high efficient parallel computation with a low external memory transfer rate could be achieved. Cheung et al. [26] surveyed the previous works using GPUs for video encoding and decoding. In addition, they presented some design consideration for GPU-based video coding.

We know that there are strong data dependencies between MBs for intraprediction. The researches on GPU-based intraprediction mainly focused on reordering the prediction modes. Kung et al. [23] and Cheung et al. [10] presented the method of reordering the process sequence of 4 × 4 blocks to increase the parallel degree. Both of their works are based on the wave-front strategy. However, limited by strong data dependence, the parallel degree is not high. Even worse, the initialized parallel degree is very low when using wave-front method. For 1080 p video format, the average parallel degree is less than 128. Ren et al. [37] presented a streaming parallel intraprediction method based on stream processor.

The research about parallelizing CAVLC and deblocking filter is very little. As control intensive components of video coding, they post a challenge to parallelize these two algorithms on massively parallel architecture efficiently. Pieters et al. proposed a deblocking filter based on GPU [24], by introducing the limited error propagation effect [38], which can filter the MBs independently. Zhang et al. [29] presented an efficient parallel framework for deblocking filter based on many-core platform, which divided the deblocking filter into two parts and used a Markov empirical transition probability matrix and a Huffman tree to further accelerate the process. To the best of our knowledge, there is no GPU-based CAVLC implementation before our work. In [39], it presented a DSP-based implementation of CAVLC. Xiao and Baas [25] proposed a parallel CAVLC encoder on fine-grained multicore system. A streaming CAVLC algorithm was described in [14].

Though a lot of works focused on accelerating various modules of H.264 encoder with GPU, as far as we know, none of them implemented the whole H.264 application on GPU, except the CUDA encoder. We think that it is difficult to efficiently parallelize the H.264 encoder based on GPU for four reasons. First, H.264 encoder itself is a very complex application due to high computation requirement and frequent memory access [40]; second, the gap between the traditional serial H.264 framework and the massively parallel architecture, which makes it difficult to implement H.264 on GPU. In the traditional program of H.264, a video frame is processed MB by MB sequentially. The granularity is very small, 256 bytes, which is violated with the massively parallel mechanism of GPU. Furthermore, CAVLC and deblocking filter, consisting of irregular computation and random memory access [14, 29], pose a challenge to GPU programming. Finally, the data transfer between CPU and GPU could be one of the major bottlenecks for achieving high performance. Taking the 1080 p video format as an example, the data size needed to be transferred is more than 30 megabytes. For the PCI-E bus 2.0, the peak bandwidth is 8 GB/s; assuming the transfer efficiency is about 40%, the data transformation time is more than 10 ms. Actually, the total 30 megabytes data is transferred by many times, and memory copy startup overhead should be considered.

## 3. The Proposed Parallel Framework

### 3.1. Profiling the H.264/AVC

H.264 video coding standard is designed based on the block-based hybrid video coding approach [1, 13]. It mainly includes four parts, from interprediction, intraprediction, and entropy encoding to deblocking filter. In this paper, we choose x264 program as reference code to analyze the feature of H.264 encoder.  Figure 1 shows the skeleton of the x264 encoder. It can be seen that the program is organized by triple loops: MB, slice, and frames. A frame is divided into many 16 × 16 MBs. The whole frame is processed MB by MB in raster order, from prediction to CAVLC. Obviously, this kind of program structure is not fit for GPU-like parallel platform in several aspects. First, the process granularity is too small. The granularity of the H.264/AVC is one MB (256 pixels), while the number of processor units of modern GPU is more than 300. Second, the process path is too long to parallelize. The number of instructions between two iterations is more than one million [40]. In addition, the essential functions, such as  sub4 × 4_dct(), are nested deeply, which increases the complexity of kernel designing.

### 3.2. Loop Partitioning in terms of Frame

In order to map the H.264/AVC program onto GPU, we firstly optimized the structure of the x264. The loop partition technology is adopted to divide the long path into several short ones, as shown in Figure 2. The functions are segmented in terms of frame. For a frame, it performs the interprediction for all MBs firstly. After the prediction of all the MBs is finished, the other functions can begin to execute on the MBs. Though much larger memory space is needed to keep the temporal data, it makes the parallel designing simplify. The programmer can focus on paralleling each individual module.

### 3.3. Data Locality: From AOS to SOA

There are lots of large data structures in x264 procedure, such as MB_INFO, which integrates the common information of a MB, shown in Algorithm 1. Each instance of this data structure needs a memory space with size of 52 (13 × 4) bytes. However, each access to the structure only requires one or several of its elements. For example, only 4 elements are typically used in intraprediction, while the amount of data involved is 52 × #*MBs* (number of macroblocks) bytes. The bandwidth efficiency is only 4/13. In addition, adjacent threads of a kernel usually access the same continuous elements of MB_INFO. For example, assume that thread 0 accesses the motion vector (MV in the MB_INFO structure) of MB1, and there is a high probability that thread 1 will accesses the MV of MB2. However, the access stride of each thread is 52 bytes. When loading from global memory, the sustained bandwidth efficiency is only about 1/13.

In order to improve the bandwidth efficiency, a transformation from AOS to SOA was performed. Corresponding to decoupled kernels, large global data structures are converted into many small local data structures. Which brings the following three advantages. (1) It improves the data transfer efficiency by avoiding unnecessary data loading. For example, in the intraprediction process, the 4 parameters loaded are valid. (2) It improves data locality, facilitating prefetching. (3) It facilitates coalesced access to GPU memory, which uses the available memory bandwidth more efficiently.

### 3.4. Offloading the Workloads to GPU

Besides the compute intensive tools, there are also control intensive components in the H.264/AVC, such as CAVLC and deblocking filter. The execution time for these two parts takes about 20% of the total time. If these components cannot be parallelized efficiently, the performance of parallel H.264 encoder will be restricted by the serial parts. In this paper, we decomposed the H.264 encoder according to the functional modules into multi-independent tools. These tools are connected according to the input and output relationship. We assigned all the major workloads of H.264 encoder to GPU, while the CPU is just responsible for some simple transactions, like I/O. The proposed H.264 encoder architecture based on GPU is presented in Figure 3. The optimized structure takes on the following characteristics. The first one is the relatively independent functional modules, which handle large volumes of data with multiple loops. It implies rich parallelism if loop unrolling is available. The other one is the locality of the producer-consumer. This feature can reduce the data transfer between CPU and GPU. However, the challenges generated from parallelizing the control intensive components (CAVLC and deblocking filter) still exist in this framework. In fact, it must modify the corresponding algorithms to settle this kind of problems, which will be discussed in the following sections.

## 4. MRMW: A Scalable Parallel Motion Estimation Algorithm

Motion estimation typically consists of two parts, the calculation of the sum of the absolute difference (SAD) for each possible estimate mode and the evaluation of rate-distortion (RD) performance of each mode. It is the most time-consuming part of video encoder [9]. In addition, the process for RD evaluation may restrict the parallel degree. In this paper, a novel ME algorithm is proposed, named multiresolutions multiwindows (MRMW) motion estimation. The basic idea of MRMW is using the motion trend of a lower resolution frame to estimate that of the original frame. It firstly compacts the original frame into lower resolution image and estimates a primary MV for each compacted MB. Based on the generated MV, it calculates a refinement MV of MB in the original frame. The algorithm is divided into three stages as follows.

Generating lower resolution frames: taking the 1080 p video format as an example, the resolution (1920 × 1080) image is decimated to a half-resolution (960 × 540) image and a quarter-resolution (480 × 270) one, shown as in Figure 4. The sizes of concentrated MB are 8 × 8 and 4 × 4 for half-resolution and quarter-resolution images, respectively.

Full search on low resolution images: in order to ensure the accuracy of the search results, a large search window is assigned, such as 32 × 32. That is to say, when extended to the original 1080 p resolution, the search window space covers a 128 × 128 region. Through this way, a rough MV is generated for each MB, which is the candidate holding the minimal SAD value, shown as in Figure 4, named MV0. Then, a similar search process is performed in a small window space for MBs in the half-resolution frame. The search window is centered with MV0. In this step, a more accurate MV is generated, named MV1 in Figure 4. In addition, we divided the whole frame into several independent tiles to enlarge the parallel degree, similar to the tiles of HEVC. The process to MBs in different tiles can be executed simultaneously.

Refinement search for full-resolution: it calculates a MV for each MB in the original frame like the process to MB of the half-resolution. Then, an evaluation of rate-distortion performance is performed to generate the final optimal MV. It should be noticed that we considered the whole frame as only one tile in this step. In order to obtain a more accurate prediction result, a MB is divided into variable block sizes, such as 8 × 4, 4 × 8, 8 × 8, 16 × 8, 8 × 16, and 16 × 16. If the estimation is processed for each kind of block, the MV would be the most accurate. However, the computation requirement will be the highest. In this paper, the SAD values of different blocks are merged from the corresponding 4 × 4 subblocks' values.

All three steps of MRMW consist of the following two basic functions: computing SADs for each candidate position and selecting the best MV. In order to maximize the parallelism, we divided each step of MRMW into three stages: the computation of SADs, merging of SADs, selection of the best MV. In this section, the processing for the full-resolution is chosen to explain the parallel implementation of the proposed interprediction algorithm with CUDA.

In our implementation, a MB was divided into 16 subblocks with size of 4 × 4. The SAD value of each 4 × 4 subblock can be calculated simultaneously for all search points. Using the generated SAD values of 4 × 4 subblocks, the SAD value for other sizes of block can be calculated. One thread is assigned to process the computation for a candidate search point. Assuming the search range is *M* × *N*, the number of thread of the kernel can be computed by (1). Because there are two iterations of similar operations that will be carried out before processing the full-resolution frame, we assigned the search range as 16 × 16 for saving computation. For 720 p, the parallel degree achieves up to 14745600. Assuming the size of the thread-block is 256, the total number of thread-block achieves 57600, while the number of multi-stream-processor (SM) in a GPU graphic is less than 50. That is to say the number of thread-block assigned to each SM is more than 1000.  Figure 5 shows the parallel model of SAD computing based on CUDA. Each thread calculates the SAD value for a 4 × 4 subblock in a certain search position. A thread-block deals with computation for a 4 × 4 subblock in the same search window (20 pixels × 20 pixels). In order to reduce the accessing to global memory, the pixels of a search window are loaded to the shared memory and can be reused by all threads of the same thread-block.  Figure 6 shows the course of merging SAD. Firstly, the SAD values of small blocks (4 × 8 and 8 × 4) are obtained. Then results for big blocks will be produced based on the small ones. The kernel designation is different from SAD computation; one thread corresponds to one MB, but not the subblock:

(1) $$\begin{array}{c} {\text{Num}}_{\text{thread}}=\frac{\text{width}}{4}\times \frac{\text{height}}{4}\times N\times M. \end{array}$$

## 5. Efficient Parallel Designs for Control Intensive Modules

### 5.1. Multilevel Parallelism for Intracoding

#### 5.1.1. Dependence Analysis

Two kinds of intraprediction are largely used for component of Luma coefficient: the 4 × 4 mode and the 16 × 16 mode. The 4 × 4 prediction pattern contains 9 methods [1]. Similarly, there are 4 methods for the 16 × 16 mode. For each mode, reconstructed pixels in neighbor blocks or MBs are needed, which makes the process of current MB must wait until its left-top MB, top MB, and left MB are completely performed. This kind of dependence severely restricts the parallelism of intracoding.

#### 5.1.2. Exploring the Parallelism between MBs

In order to increase the parallel degree, multislice method is introduced. It partitioned each frame into multislice and processed each slice independently. At the same time, the wave-front method is adopted for parallelizing the MBs in the same slice, shown as in Figures 7(a) and 7(b). It should be noticed that multislices will also result in the reduction of the compression rate. However, if the number of slices is kept within a small value, such as 17 for 1080 p video format, the experimental results show that the reduction of the compression rate is acceptable.

#### 5.1.3. Exploiting the Parallelism within a MB

Restricted to the reconstructed loop, though adopting wave-front method, ten steps are needed to accomplish the 4 × 4 mode prediction for a MB. As is shown in Figure 7(c), here, each small grid represents a 4 × 4 block. The number indicates the encoding order of the blocks. The arrow represents data dependence. From the graph, we know that the maximal number of blocks within a MB that can be performed simultaneously is only 2. Experiments to multiple test sequences show that some prediction methods, needing upper right reconstructed pixels (the third and the seventh method of the 4 × 4 prediction and the third of the 16 × 16 prediction), play a slight role. It increases the bit-rate for I-frames by less than 1% and has an even smaller impact on P-frames when dropping these three prediction ways. Therefore, in this paper, we remove these three modes. Figure 7(c) shows that the intracoding of a MB can be completed in 7 steps and the parallel degree can reach 4 for a MB. After optimizing with the above two steps, the total max parallel degree for intraprediction achieves 272 for 1080 p video format, when the slice number is configured as 17.

#### 5.1.4. Maximal Parallelism of the Pipeline

We divided intracoding into five stages: prediction, DCT, quantization, I_quantization, and IDCT. The granularity of data dependency in a MB differs from various stages, shown as in Table 1. This feature induces us to design parallel model according to different stages. We first configure thread-block according to the available maximum parallel degree. During execution, states of a thread are variational with different stages. For a MB with size of 256, the maximum number of threads that can be executed simultaneously is 256 in stage of quantization, so the size of thread-block will be set as 256. In prediction stage, only 16 threads are activated for each thread-block. During the processing of DCT, 64 threads work and each thread handles a row/column of pixels in a 4 × 4 block. When coming into quantization phase, all threads are activated. Experimental results show that the multilevel parallel method can achieve 3 times the speedup ratio compared with using constant parallel degree.

### 5.2. Component-Based Parallel CAVLC

#### 5.2.1. Three Major Dependencies of CAVLC

Through profiling the instructions of CAVLC, we found three major factors that restrict its parallelism, that is, the context-based data dependence, the memory accessing dependence, and the control dependence. Context-based data dependence is caused by the self-adaptive feature of CAVLC, shown as in Figure 8(a). The value of nC of the current block relies on nA and nB. Due to the dependence, the process to current block must wait until its top block and left block are finished. The memory accessing dependence is due to the variable length coding characteristic of CAVLC, shown as Figure 8(b). As we all know, the bit-stream of a frame is packed bit by bit, and the bit-stream of current MB cannot be output until the prior one is performed. Control dependence results from different processing path for different components, which consists of two layers: the frame layer and the block layer. In the frame layer, the branch is mainly caused by different frame types and different components of a frame. The left side of Figure 8(c) describes the branch caused by computing the value of nC for different component block. In the block layer, the branch comes from the irregular characteristic of symbol data, such as whether sign_trail is 1 or −1 and whether levels are zero or not. The right side of Figure 8(c) gives the branch processes of computing the symbol of levels.

In order to parallelize the CAVLC encoder on GPU, the first step is to optimize the structure of the conventional CAVLC to overcome the limitations described above. We partitioned the CAVLC into four paths according to the four components of a frame: Luma_AC, Luma_DC, Chroma_AC, and Chroma_DC. For each processing path, three stages are performed, that is, coefficient scan, symbol coding, and bit-stream output. The proposed CAVLC encoder, named component-based CAVLC, is shown in Figure 9.

#### 5.2.2. Two Scans for Data Dependence

Two scans are employed to gain the statistic symbols. Firstly, a forward scan is executed on the quantized residual data, and it stored the residual data in zigzag order. The results include the number of nonzero coefficients (total_coeff: nA/nB) of blocks and the zigzagged coefficients. Then, a backward scan is performed on the zigzagged coefficients. According to the value of nA/nB, the value of nC can be calculated. The results consist of symbols needed to be coded and the values of nC. This method wins two advantages: avoiding data dependence when computing nC and reducing unordered memory accessing for zigzag scan in the traditional codes.

#### 5.2.3. Component-Based Parallel Coding

For the sake of minimizing the performance loss of the target parallel CAVLC encoder due to control dependence, in this paper, we proposed a component-based coding mechanism. In this method, the program codes the symbols frame by frame in order of Luma_DC, Luma_AC, Chroma_DC, Chroma_AC, instead of processing the four components MB by MB. For example, until all the coefficients of Luma_DC of a frame are executed, the process for the component of Luma_AC could be started. The unnecessary branches caused by different process path can be effectively reduced. In this stage, the coded results (the bit-stream for each symbol and its length) must be kept for the next stage (packing). However, the size of bit-stream of each block is unknown; a big enough temporary memory space is required to store the corresponding bit-streams. In our implementation, maximum of 104 bytes are used for keeping the symbols of a subblock. It should be noticed that, among those memory units, some of them are not used.

#### 5.2.4. Parallel Packing

In order to implement the parallel packing, the behavior of each thread must be determinate. It means that the output position of the bit-stream for each block must be determinate. Though the length of the bit-stream is not constant, fortunately, the length of bit-stream of each block has to be obtained from the previous stage. According to the length, the output position can be calculated for each subblock and a parallel packing can be performed. In this paper, two steps are employed to perform the parallel packing. The first step combines the bit-stream of subblocks of a MB to be a continuous one and computes the parameters for parallel packing, which includes the out position, the shift bits, and shift mode of the bit-stream for each MB. The second step performs parallel packing based on the parameters gained in the first step.

We firstly combine the bit-stream of each subblock to be a continuous one. For this kernel, the number of thread is equal to the number of blocks of a frame. Then, it packs the bit-stream of different blocks of an MB to form an integrated one. The number of threads reduces to be the number of MB. In order to parallelize the packing for each MB, some information is needed, shown as follows:

- the number of byte of bit-stream for each MB (*n*);
- the number of the remaining bits less than one byte of the bit-stream for each MB (*m*, *m* < 8);
- the shift mode and shift bits for the bit-stream of each MB.

The length of bit-stream for each MB is (*n* × 8 + *m*) bits. According to the length, the output position of the bit-stream for each MB can be obtained. The reduce method is adopted to speed up the calculation, shown as in Figure 10.

In the second step, each thread disposes the writing back process of bit-stream for one MB. In our implementation, a composed byte is generated by shifting the current bit-stream towards left and the next bit-stream towards right. The shifted number is 8 m for left-shift and *m* for right-shift, respectively.  Figure 11 shows the progressing of parallel output. In the first writing, thread T0 writes the first byte of the bit-stream of MB0. Thread T1 writes the composed byte of MB1, which is the combination of the last two bits of the first byte and the first six bits of the second byte of the bit-stream. The data thread T0 writing in the last time is a composite byte of the last two bits of MB0 and the first six bits of MB1.

### 5.3. Direction-Priority Parallel for Deblocking Filter

#### 5.3.1. Dependence Analysis

Deblocking filter is performed to eliminate the artifacts produced by block-based coding. For a frame, each MB is filtered in raster-scan order with optional boundary strength (BS). The filter order for edges of luminance MB is shown in Figure 12. The program firstly filters the vertical boundaries from left to right (from A to D), followed by four horizontal boundaries (from E to H). For chrominance MB, it filters the external boundary of the MB followed by the internal boundary. The filtering to edges of the current boundary (such as e5, e6, e7, and e8 of B Figure 12) depends on the results of the edges of the previous boundary (e1, e2, e3, and e4 of edge A in Figure 12). Similarly, the process to the current MB must wait until the previous one is finished. It is challenging to parallelize deblocking filtering efficiently due to this dependence.  Table 2 shows the performance of serial implementation on CPU and a nonoptimized parallel one on GPU GTX260. The performance of the parallel realization is 4.4 times lower than that of the serial one. The major reason can be attributed to the very small parallel degree.

#### 5.3.2. Direction-Priority Algorithm for Filter

Through the analysis to the instructions, we found that the difference between the filtered pixels and the original pixels is very small. In addition, data dependence between MBs only involves the outermost boundaries. Furthermore, the dependence level varies from the BS. Based on the observation, in this paper, to enlarge the degree of parallelism, a direction-priority deblocking filter was proposed, shown as Figure 13. The process of the proposed algorithm is as follows: filtering pixels around vertical edges of the frame from left to right followed by filtering pixels around horizontal edges of the frame in top-to-bottom order. Different from MB-based approach [10], the direction-priority approach decouples the computations for different directions. Each thread of the kernel processes a pixel and the surrounding pixels on the same edge, so that pixel-level parallelism can be achieved. In this way, the highest degree of parallelism for vertical filtering is 1088, while horizontal filtering achieves 1920.

#### 5.3.3. Four Steps Schedule to Enlarge the Parallel Degree

In order to further explore the parallelism, we proposed a novel schedule method. The processing for a MB is divided into four steps according to the principle of the limited error propagation [38]. During each step, the filter to all MBs is independent, but explicit synchronization is necessary for neighboring steps.  Figure 14 shows the proposed schedule strategy. As we know, the strong filter just exists at the boundaries of MB (boundary 0 or boundary 4 in Figure 14(a)). For the inner boundaries (boundaries 1, 2, and 3 and boundaries 5, 6, and 7), maximal two pixels on either side of the boundaries may be affected. For example, the samples (g, h, and i) used for filtering the second pixel of the right side of the boundary 2 (pixels j) will not be affected, shown as Figure 14(a). Based on the above analysis, the proposed scheduling is shown as follows: in the first step, a horizontal filtering to samples of boundary 2 and boundary 3 (samples from j to n) is performed for all the MBs. Five columns pixels will be modified, shown in Figure 14(a). The pixels of other columns (pixels: n p and a i) will be filtered in horizontal way in the second stage in Figure 14(b). Similarly, a vertical filter is carried out for the horizontal boundaries (boundary 6 and boundary 7) in step three, shown as Figure 14(c), and the pixels rows from J to M will reach their final state. In the final stage, the pixels from N to P and from A to I of a MB are filtered in Figure 14(d). At the start of the second step, a synchronization point is introduced to ensure that the horizontal filter for boundary 3 of the previous MB is finished.

Through the two steps mentioned above, the parallel degree of the deblocking filtering is increased significantly.  Table 3 shows the parallelism of the conventional algorithm and the proposed algorithm. It can be seen that the parallelism is always 16 for serial algorithm, while the parallelism of the proposed method increases with the resolution of the video.

## 6. Experimental Results and Analysis

### 6.1. Experimental Setup and Test Sequences

The proposed parallel H.264 encoder was tested on the host of Alienware Aurora-R3, which was equipped with Intel CPU i7-2600 (quad-core 3.4 GHz). Three different NVIDIA GPUs are chosen as coprocessors to accelerate the proposed parallel H.264 encoder. The detailed information of the GPUs can be seen in Table 4. The CUDA used in our experiment was CUDA-4.2. The input videos in our experiment consist of a list of standard test sequences in three resolutions: D1 (City, Crew), 720 p (Mabcal, Park_run, Shields, and Stock), and 1080 p (Into_tree, Old_town, Park_joy, and Rush_hour).

### 6.2. Evaluation of the RD Performance

We first evaluated the RD performance of the proposed parallel H.264 encoder.  Figure 15 shows the detailed impacts of different algorithms on RD performance. The item of* Original* means the results of the reference x264 code. The* Para. Inter* represents using the proposed MRMW algorithm instead of the original ME in x264 and keep the other components unchanged, while* Para. Intra* and* Para. DB.* mean introducing the proposed multilevel parallel intracoding and the direction-priority deblocking filter to x264 code, respectively. The* Para. App.* presents the implemented CUDA-based parallel H.264 encoder. Because we do not propose a new CAVLC algorithm, but just reorder the execution sequence, there is no impact to the RD performance. The tested sequences are configured as P-frames followed with an I-frame for each 30 frames. All the sequences are encoded for total 300 frames. The slice numbers are set as 11, 15, and 17 for video formats of D1, 720 p, and 1080 p, respectively. The initial search range for MRMW is 16 × 16. It can be seen that the degradations of PSNR are from 0.08 dB to 0.56 dB compared with the reference software, when using the MRMW algorithm. The decrease of the PSNR can be attributed to the following two reasons. The first one is that the proposed MRMW algorithm divided the whole frame into several small subdomains, which is a 2D grid and consists of several MBs. The ME is independent for each subdomain. In addition, the MV of compacted lower-resolution MB may not represent the real MV of the original MB. The decline of the PSNR values affected by multilevel parallel intracoding is less than 0.1 dB for 1080 p, when keeping the same bitrate. For the other two formats of frames, the maximal degradations of PSNR are 0.19 dB and 0.32 dB, when the bitrate is about 3000 kbps. With the bitrate increasing, the degradation of PSNR impacted by multilevel parallel intra-algorithms is decreasing. When the bitrate is larger than 20000 kbps, the degradations of PSNR are smaller than 0.08 dB, while for the direction-priority deblocking filter, the impact to RD-performance could be negligible, and results show upgrades in some cases even. Overall, compared with the reference program, the implemented CUDA H.264 has a loss of PSNR value about 0.35 dB ~ 0.54 dB, 0.14 dB ~ 0.77 dB, and 0.33 dB ~ 0.57 dB for D1, 720 p, and 1080 p video formats, respectively.

### 6.3. The Speedup Overhead Analysis

We then assessed the speedup of the proposed encoder. Figures 16, 17, and 18 give the speedup ratio of the CUDA-based H.264 encoder on three NVIDIA's GPUs, compared with the performance of the serial program on Intel CPU i7-2600. It should be noticed that the serial program was not optimized with vectorization. The experimental results indicate that our implementation outperforms the reference serial encoder in terms of speedup ratio by a factor of more than 19 for 1080 p format on C2050. For the performance on GTX460 and GTX260, the speedup ratios of the application are about 16 and 11. One observation is that the bigger the input sequences, the higher the speedup ratio that can be achieved. Except the overall performance of the H.264 encoder, we also evaluated the performance of different parallel components. From the graph, it can be seen that the interprediction achieves the maximal speedup. The speedup ratios on three GPUs are about 13, 18, and 25, respectively. We considered that the high speedup ratio comes from the high parallel degree of the MRMW. We noticed that the achieved speedup ratios are proportional with the peak performance of the GPUs. It implies that the proposed MRMW algorithm is scalable, while for intraprediction, the speedup ratio is very low, about from 2.8 to 8.8. That is because of the strong data dependence caused by the reconstruction loop, which is suitable for execution on CPU. For the control intensive components CAVLC, the speedup ratios on the three platforms are similar to each other and are proportional with the memory bandwidth, while deblocking filter shows varied phenomenon, because the parallel degree of the most time consuming kernel (bit_pact) of CAVLC is relatively small and decreases with the kernel execution. Moreover, the process of this kernel is irregular, which cannot exploit the computational power of GPUs. In addition, the computation-accessing-ratio of CAVLC is relatively low; the performance of the proposed CAVLC is majorly determined by the bandwidth of the GPU, while the parallel degree of the proposed deblocking filter is equal to the number of 4 × 4 subblock of a frame and keeps constant during the kernel execution. It should be noticed that the CAVLC achieves a very high performance on the CPU used in this paper due to its high frequency and big cache size. When compared with the performance on another CPU, Intel E8200, the speedup ratio of CAVLC can be 46, 4 times higher than the speedup on Intel CPU i7-2600.

We also compared the performance of the proposed parallel implementation of H.264 encoder with other versions based on GPU or multicore processors, shown as in Table 5. As can be seen, our implementation can achieve about 16 times of speedup compared with the reference program without optimization for 720 p. It outperforms the optimized serial encoder (using compiled instructions, MMX, SSE, and so on) in term of speedup by factors from 3 to 6. It should be noticed that the speedup ratios in the table for other implementations are copied from the corresponding papers, but not the results compared with the performance tested on our CPU. In order to facilitate comparison with other GPU-based implementations, we list the performance of different modules on GTX260. A significant improvement can be obtained for the proposed encoder when compared with other GPU-based parallel versions. Our implementation establishes a speedup factor of 3 over the parallel H.264 encoder based on GPU [10]. More than 5 times of speedup can be achieved for the proposed multilevel intracoding compared with the wavefront method [23] for 720 p video pictures, when normalized to the same reference CPU. This table clearly shows that our component-based CAVLC outperforms the implementation based on fine-grained multiprocessors system [25]. For deblocking filter, we got a similar speedup with MFP [24]. For 720 p format scenarios, the proposed parallel H.264 encoder can satisfy the requirement of real-time encoding of 30 fps, while for 1080 p, the encoding speed achieves 20 fps. We think two major factors make the proposed encoder high performance. The first one is that the implementation realizes all the major workload of the H.264 encoder with GPU, even for the irregular components. It eliminates the impact of serial parts according to Amdahl's low and reduces the cost of data transfer between CPU and GPU. The other one is the proposed novel algorithms for varied modules, which enlarge the parallel degree as much as possible and improve the efficiency of the memory bandwidth. Though the CUDA encoder can achieve a better performance on speedup ratio, the quality is not as good as the proposed implementation. More importantly, there is no detailed information about the designation of the CUDA encoder.

### 6.4. The Bottleneck Analysis

In this section, we discuss the time breakdown of the proposed H.264 encoder.  Figure 19 shows the time distribution of the parallel H.264 encoder on different platforms, including the CPU. As can be seen, the inter prediction occupies more than 70% of the execution time when running on CPU. After parallelization, the proportion decreased to be about 30% on C2050. The time proportion of the parallel intraprediction doubled when compared with its result in the serial encoder. An interesting observation is that the proportion of the CAVLC rose after parallelization. In addition, the number increased with the computation power of the GPU, from 23% on GTX260 to 34% on C2050. The proportion of the deblocking filter keeps almost the same with that of the serial implementation. For the parallel implementation, though almost all the workloads are offloaded to GPU, the memory copy time consists of about 25% even.

In order to analyze the proposed H.264 encoder much more accurately, we used the CUDA profiler to collect the major metrics of kernels. The results are based on encoding 30 frames of video sequences* Shields.* Table 6 shows the detailed information of the major kernels on GTX460, including the execution time proportion, IPC, shared memory used for each thread block, the register allocated to each thread, and the performance limitation factor. Here, we just listed the information of kernels, whose execution time occupied more than 0.5% of the total execution. The Exe. time means the execution time of the kernel. The column of branch indicates the instructions executed in serial way. As can be seen, the calling times of the memory copy are 864 and 257 for host-to-device and device-to-host, respectively, we think the times of API calling caused the high proportion of these two methods. The most time consuming kernel comes from the CAVLC, named* cavlc_bitpack_block*, which packs the encoded bit-stream of each block to be a continuous one. The limitation of this kernel can be attributed to the irregular process and the calling time. We think that it is a possible optimization to packing all four kinds of bit-stream of a frame in the same kernel. Furthermore, using the L1 cache instead of the shared memory in some case may bring some benefits. Kernel* Iframe_luma_residual_coding* deals with the intraprediction, DCT, and the quantization of an I frame. Though it has been called only for one time, the time proportion is more than 5%., because the parallelism is very low, which is due to the strong data dependence. In addition, there are many branch instructions resulting from the multiprediction modes, which will cause serial execution. For most of kernels belonging to the interprediction, the performance limitation factors come from the register consuming and the parallelism. When the number of register used for each thread is over 32, the maximal occupancy that can be obtained will be less than 0.667. We also marked the kernels with lower IPC (the bold italic grids), which reveals the utilization of the compute units. The low IPC can be attributed to the serial execution and the frequent memory access. As we found from the figure, the shared memory usage will not be a performance impact factor. For some kernels that involved a lot of in/out data, the global memory of the bandwidth will restrict the performance, such as* CalcCBP_and_TotalCoeff_Luma*. It calculates the CBP coefficients and needs the transformed data as input. The data amount is double of input frame.

## 7. Conclusion and Future Work

In this paper, we proposed a parallel framework for H.264/AVC based on massively parallel architecture. Through loop partition and transformation from AOS to SOA, we optimized the program structure for parallel kernel designing. We offloaded all the computation tasks to GPU and implemented all the components with CUDA. In order to achieve high performance, we optimized all components of H.264 encoder, proposed corresponding parallel algorithms, including MRMW, multilevel parallel intracoding, component-based parallel CAVLC and direction-priority parallel deblocking filter. Particularly, in order to parallelize the control intensive parts, such as CAVLC and deblocking filter, two novel algorithms are presented. Experimental results show that about 20 times the speedup can be obtained for the proposed efficient parallel method when compared with the reference program. The presented parallel H.264 encoder can satisfy the requirement of real-time HD encoding of 30 fps. Our implementation outperforms the other GPU-based encoders in terms of speedup by factors from 3 to 10. We think there are two pivotal factors denoting the high performance of the H.264 encoder. One is the full parallel framework proposed based on multiple programmable processors. The other one is the efficient parallel algorithms for different modules.

It can be seen from the bottleneck analysis that there is rich space to optimize our implementation, such as the mechanism of stream and efficient usage of the on-chip memory, especially the L1 cache in modern GPU. With the rise of the new video coding standard H.265, we intended to parallelize it based on the technologies proposed in this paper. By paralleling this application based on GPU, we suffered from the low productivity. In the future, we are also interested in automatically parallel framework aiming at multimedia applications based on programmable multi/many core architecture.

## Figures and Tables

**Figure 1:** The skeleton of x264 program.

**Figure 2:** The loop partition of x264.

**Figure 3:** The proposed H.264 encoder framework.

**Figure 4:** Concentration of the original frame into lower resolution ones.

**Figure 5:** The parallel model for SAD computing of 4 × 4 subblocks.

**Figure 6:** The merging of SAD values for different block.

**Figure 7:** Multiple levels of parallelism of intraprediction.

**Figure 8:** Dependence of the CAVLC encoder.

**Figure 9:** The component-based CAVLC.

**Figure 10:** Calculation of start position for each MB.

**Figure 11:** Parallel writing packing.

**Figure 12:** The filtering order for boundaries of a MB.

**Figure 13:** Direction-priority approach on GPU.

**Figure 14:** Scheduling of the filter for MB.* White*: original pixels;* light gray*: previously filtered pixels;* dark gray*: filtered in current pass;* circled*: pixels in their final state.

**Figure 15:** RD performance with different algorithms.

**Figure 16:** Speedup ratio of the proposed parallel H.264 encoder on GTX260.

**Figure 17:** Speedup ratio of the proposed parallel H.264 encoder on GTX460.

**Figure 18:** Speedup ratio of the proposed parallel H.264 encoder on C2050.

**Figure 19:** Time breakdown of Shields on CPU and GPUs.

**Algorithm 1:** Structure of the MB_INFO structure in the x264 code.

**Table 1:** Characteristics of five stages.

Stages	Dependence level	Dependence granularity	Maximal parallel degree
Prediction	Strong	One 4 × 4 block	16
DCT	Weak strong	One column or row of 4 × 4 block	64
Quantization	None	One pixel	256
I_quantization	None	One pixel	256
IDCT	Weak strong	One column or row of 4 × 4 block	64

**Table 2:** The performance comparison between nonoptimized parallel deblocking filter on GPU and serial one on CPU.

Implementation	Serial	Parallel

Platform	CPU 2.65 GHz	GTX 260

Parallel degree	1	16

Performance (ms/frame 1080 p)	92.1	405.8

**Table 3:** Available parallelism of different DB algorithms.

Resolution	480 p	720 p	1080 p

Serial algorithm	16	16	16

The proposed method	1200 × 16	3600 × 16	8160 × 16

**Table 4:** The characters of GPUS.

Type	GTX 260	GTX 460	Tesla C2050

Number of SM	27	7	14

Cores	216	336	448

Frequency	1.29 GHz	1.3 GHz	1.15 GHz

Shared memory per SM	16 KB	16/48 KB	16/48 KB

Registers per SM	16384	32768	32768

L1 Cache	NA	16 KB	16 KB

Memory bandwidth	111.9 GB/s	115.2 GB/s	144 GB/s

Peak performance	535.7 Gflops	873.6 Gflops	1.03 Tflops

**Table 5:** Performance comparison between the proposed parallel H.264 encoder and other implementations.

Platform	Reference code	Target resolution	Optimized module	Speedup ratio	Performance (fps)
CPU (i7-2600) original	x264	720 p	NA	1	1.05 (for application)
CPU (i7-2600) optimized	x264	720 p	Key function	3~5	3~5.5 (for application)
GTX280 [10]	x264	720 p	ME	NA	15.5 (for ME)
Geforce 8800 [23]	x264	720 p	Intracoding	2~3	NA
AsAP [25]	x264	720 p	CAVLC	4.86	36~41.3 (for CAVLC)
GTX 240MFP [24]	x264	1080 p	Deblocking filter	10.2	1309 (for deblocking filter)
GeForce 9800 [3]	JSVM	CIF	ME + Intra	6.7	1.02 (for application)
GTX260 The proposed MRMW	x264	720 p	ME	12~14	50 (for ME)
GTX260 The proposed Intra Coding	x264	720 p	Intracoding	4~6.8	21 (for Intracoding)
GTX260 Component-based CAVLC	x264	720 p	CAVLC	8	105 (for CAVLC)
GTX260 Direction-priority DB.	x264	720 p	Deblocking filter	9	1050 (for deblocking filter)
C2050 The proposed H.264	x264	720 p	Application	13~17	32.3 (for application)

**Table 6:** Kernel information of Shields on GTX460.

Method	Number of calls	Exe. time (us)	% Exe. time	Average Value for each kernel launch				
				Branch	IPC	Shared_mem	Registers	Limited factors
memcpyHtoD	864	74184.20	**15.75% **	0.00	0.00	0.00	0.00	Number of calls
cavlc_bitpack_block	150	62971.30	**13.37% **	5215.31	***0.86***	6656.00	14.00	Parallelism
memcpyDtoH	357	60254.80	**12.80% **	0.00	0.00	0.00	0.00	Number of calls
pframe_intra_coding_luma	29	36969.20	**7.85% **	104046.00	***0.30***	3824.00	32.00	Parallelism
me_IntegerSimulsadVote	29	34574.20	**7.34% **	47548.10	***0.99***	1216.00	40.00	Registers
me_QR_LowresSearch	29	28985.80	**6.16% **	65434.90	1.36	5648.00	32.00	Registers
Iframe_luma_residual_coding	1	27286.10	**5.79% **	873822.00	1.94	5472.00	63.00	Parallelism
ChromaPFrameIntraResidualCoding	29	19010.40	**4.04% **	1895.59	***0.74***	320.00	63.00	Registers
pframe_inter_coding_luma	29	18334.80	**3.89%**	10815.80	***0.53***	1824.00	42.00	Parallelism
cavlc_texture_codes_luma_DC	90	16730.30	**3.55%**	10254.50	1.45	1008.00	18.00	Instruction issue
me_HR_Cal_Candidate_SAD	29	7972.38	1.69%	4639.97	1.25	1584.00	19.00	Block size
cavlc_block_context_iframe_LumaAC	30	7900.45	1.68%	1539.20	2.23	0.00	15.00	Instruction issue
cavlc_texture_symbols_luma_AC	30	7585.54	1.61%	23281.90	***0.94***	4096.00	23.00	Instruction issue
ChromaPFrameInterResidualCoding	29	7196.61	1.53%	7221.10	1.63	2688.00	31.00	Parallelism
me_HR_Candidate_Vote	29	6964.67	1.48%	6781.52	1.73	272.00	21.00	Parallelism
MotionCompensateChroma	29	6353.73	1.35%	4137.38	1.08	748.00	18.00	Instruction issue
memset32_aligned1D	182	4387.74	0.93%	3957.69	2.26	0.00	3.00	None
cavlc_bitpack_MB	30	4362.85	0.93%	2084.40	1.72	0.00	19.00	Global bandwidth
cavlc_block_context_PrevSkipMB	29	4307.42	0.91%	729.00	***0.79***	0.00	8.00	Parallelism
cavlc_texture_symbols_chroma_AC	30	3908.42	0.83%	9674.63	***0.40***	2560.00	22.00	Global bandwidth
me_Decimate	58	3695.84	0.78%	1345.78	1.48	512.00	13.00	Block size
CalcCBP_and_TotalCoeff_Luma	30	3498.78	0.74%	257.47	1.63	4608.00	21.00	Global bandwidth
CalcPredictedMVRef	29	3313.12	0.70%	230.28	1.45	0.00	18.00	Parallelism
CalcCBP_and_TotalCoeff_Chroma	30	2855.01	0.61%	1148.83	***0.82***	2528.00	23.00	Global bandwidth
cudaDeblockMB_kernel_ver	30	2851.80	0.61%	35558.30	1.19	1040.00	31.00	Global bandwidth
cavlc_block_context_ChromaAC	30	2764.67	0.59%	643.33	1.82	0.00	27.00	Registers
